The article "An Enhancement on Convolutional Artificial Intelligent Based Diagnosis for Skin Disease Using Nanotechnology Sensors" was retracted in 2023. Reasons: signs of a paper mill; suspected computer-generated content; unreliable results or conclusions; concerns about the data.

# An Enhancement on Convolutional Artificial Intelligent Based Diagnosis for Skin Disease Using Nanotechnology Sensors

**DOI:** 10.1155/2022/9539503

**Published:** 2022-07-04

**Authors:** Dr Aruna R, Srihari K, Dr Surendran S, Jagadeesan S, Somasundaram K, Dr Yuvaraj N, Deepa S, Udayakumar E, Shanmuganathan V K, Chandragandhi S, Baru Debtera

**Affiliations:** ^1^Department of Computer Science and Engineering, School of Computing, Vel Tech Rangarajan Dr Sangunthala R &D Institute of Science and Technology, Chennai, India; ^2^Department of Computer Science and Engineering, SNS College of Technology, Coimbatore, India; ^3^Department of Computer Science and Engineering, Tagore Engineering College, Chennai, TamilNadu -600 127, India; ^4^Department of Computer Science and Engineering, Vel Tech Rangarajan Dr.Sagunthala R&D Institute of Science and Technology, Avadi, Chennai, India; ^5^Department of Information Technology, Saveetha School of Engineering, SIMATS, Chennai, India; ^6^Research and Publications, ICT Academy, IIT Madras Research Park, Chennai, India; ^7^Department of Computer Science Engineering, KIT-Kalaignarkarunanidhi Institute of Technology, Coimbatore, India; ^8^Department of Electronics and Communication Engineering, KIT-Kalaignarkarunanidhi Institute of Technology, Coimbatore, India; ^9^Department of Mechanical Engineering, J.N.N Institute of Engineering, Kannigaipair, India; ^10^Department of Computer Science and Engineering, JCT College of Engineering and Technology, Coimbatore, India; ^11^Department of Chemical Engineering, College of Biological and Chemical Engineering, Addis Ababa Science and Technology University, Addis Ababa, Ethiopia

## Abstract

Skin disease is the major health problem around the world. The diagnosis of skin disease remains a challenge to dermatologist profession particularly in the detection, evaluation, and management. Health data are very large and complex due to this processing of data using traditional data processing techniques is very difficult. In this paper, to ease the complexity while processing the inputs, we use multilayered perceptron with backpropagation neural networks (MLP-BPNN). The image is collected from the devices that contain nanotechnology sensors, which is the state-of-art in the proposed model. The nanotechnology sensors sense the skin for its chemical, physical, and biological conditions with better detection specificity, sensitivity, and multiplexing ability to acquire the image for optimal classification. The MLP-BPNN technique is used to envisage the future result of disease type effectively. By using the above MLP-BPNN technique, it is easy to predict the skin diseases such as melanoma, nevus, psoriasis, and seborrheic keratosis.

The article "An Enhancement on Convolutional Artificial Intelligent Based Diagnosis for Skin Disease Using Nanotechnology Sensors" was retracted in 2023. Reasons: signs of a paper mill; suspected computer-generated content; unreliable results or conclusions; concerns about the data.

## 1. Introduction

Skin disease: skin illness is the fifth driving motivation behind death on the planet during the most recent long term. As per the World Health Organization (WHO) record, skin issue is the main rationale of death across the world representing 1.58 million, everything being equal. Early location of skin sickness is fundamental in bringing down presence misfortunes [1]. Whenever neglected to analyze the skin infection type in a beginning phase, it will prompt skin malignancy and furthermore even to death. Early location of skin sickness is fundamental in diminishing life misfortunes. Anyway, prior treatment requires the capacity to identify skin illness in beginning phases. Early analysis requires an exact and solid determination system that permits doctors to recognize amiable skin cancer from dangerous ones [2]. The fundamental point of this investigation is to perform various sorts of skin sickness images are bunch together in informational index and prepreparing the info image utilizing convolutional artificial intelligence (CAI) [3] which is a deep learning (DL) calculation to discover the kind of skin illness. Image preprocessing incorporates three significant advances that are data cleaning, data decrease, and data change. The machine or deep learning algorithm suffers mostly from the problem of overfitting due to large number of training data. In order to resolve this, the study uses BPNN model to reduce the problem of overfitting.

A multilayered perceptron–backpropagation neural network (MLP-BPNN) which is a deep learning algorithm used to diagnose the disease affected by the person. The image processing techniques are used for processing the images and storing the datasets. Those data sets will be processed apparently for classification and will be used when it is required for comparative checking of the given input from the user. This is based on the machine learning algorithms that are used for solving the comparison [4]. MLP-BPNN algorithm is the main role in departing the output for the specific input. Based on this output which is generated from the given input, the image processing gets compiled with the classification of huge data sets and then comes into the conclusion of output.

The main contribution of the work involves the collection of images from nanosensors, which is the state-of-art in the proposed model. The nanotechnology sensors sense the skin for its chemical, physical, and biological conditions with better detection specificity, sensitivity, and multiplexing ability to acquire the image for optimal classification.

## 2. Related Works

Cancer recognizable proof and expectation are immense test to the specialists (Pallavi and Prasanna [5]) . The utilization of different methods of information mining strategies has reformed the entire cycle of malignant growth diagnosis and prognosis [6]. We are proposing coordinated framework which depends on mix of different information mining methods, for example, logical chain of command measure, rule-based affiliation, and arrangement that is useful to anticipate the patient's infection status. Malignancy sickness danger can be found by investigating and recognizing different components and manifestations of the patient prior to suggesting therapies [7]. The crucial point of our framework is to help oncologist and clinical specialists in diagnosing the patient by breaking down accessible information and important data [8]. Krishnaiah et al. [2] proposed the classification using rule mining and Naïve Bayes to support the medical services. The Bayes classifier is used to preprocess and feature extract the instances in a better manner [9].

The article "An Enhancement on Convolutional Artificial Intelligent Based Diagnosis for Skin Disease Using Nanotechnology Sensors" was retracted in 2023. Reasons: signs of a paper mill; suspected computer-generated content; unreliable results or conclusions; concerns about the data.

Information mining is characterized as filtering through a lot of information for valuable data (Sudha and VijayaraniJan [10]). The absolute generally significant and well-known information mining procedures are affiliation rules, characterization, grouping, expectation, and consecutive examples. Information digging strategies are utilized for assortment of uses. In medical care industry, information mining assumes a significant part for anticipating sicknesses. For recognizing an infection, number of tests ought to be needed from the patient. But, for utilizing information mining procedure, the quantity of test ought to be diminished [11]. Karthikeyan and Thangaraju [12] introduced an extraction calculation used to improve the anticipated precision of the order. This paper applies with principal component investigation as an element evaluator and ranker for looking through strategy. Innocent Bayes calculation is utilized as an arrangement calculation. It dissects the hepatitis patients from the UCI AI archive. The aftereffects of the characterization model are exactness and time. At last, it infers that the proposed PCA-NB calculation execution is superior to other characterization methods for hepatitis patients.

These days individuals work on PCs for quite a long time they do not have the opportunity to deal with themselves (RuchaShinde and PriyankaPatil [13]). Because of frenzied timetables and utilization of shoddy nourishment, it influences the soundness of individuals and principally heart. So, we are actualizing a coronary illness expectation framework utilizing information mining method Naïve Bayes and k-implies grouping calculation. It is the blend of both the calculations. This paper gives a diagram for the equivalent. It helps in anticipating the coronary illness utilizing different ascribes, and it predicts the yield as in the expectation structure. For gathering of different ascribes, it utilizes k-implies calculation, and for anticipating, it utilizes innocent Bayes calculation [2]. Mugdha S Manerkar et al. utilize C methods and Watershed calculations for image division. Highlight extraction is performed utilizing gray-level cooccurrence matrix (GLCM) and image quality assessment (IQA) techniques for surface which gave the measurable boundaries of every calculation, features benefits of preparing information and testing [14]. G. Ramya and J. Rajeshkumar utilized GLCM strategy for separating highlights from the fragmented ailing and grouped the skin malignancies dependent on fluffy arrangement, higher precision contrasted with existing one.

The article "An Enhancement on Convolutional Artificial Intelligent Based Diagnosis for Skin Disease Using Nanotechnology Sensors" was retracted in 2023. Reasons: signs of a paper mill; suspected computer-generated content; unreliable results or conclusions; concerns about the data.

Nanosensors [15–19] can be used in a variety of ways. For environmental agencies, the capacity to detect biological agents in water and air is an issue. Because of their small size, speed, and accuracy, nanosensors will revolutionise air and water quality monitoring.

New methods for air sampling are being developed that use nanosensors for the detection of quality of air, especially on contaminants. Researchers in East Asia and the Pacific have employed nanosensors to study aerosol interaction and irradiance in the region.

This kind of equipment has proven effective for monitoring the level of air pollution at Beijing. An Israeli start-up business will utilize nanosensors to monitor and analyze automobile engine emissions to meet the increasingly severe regulations of environmental agencies.

Additionally, nanosensors can be utilized to keep tabs on things like water distribution and quality. The Environmental Protection Agency has created a cost-effective monitoring system to repair the water supply infrastructure due to faulty pipes and mains. Using nanosensors, this “Smart Pipe” prototype will keep tabs on water flow and quality.

Without changing the existing infrastructure's flow conditions, it will be possible to monitor flow rates in real time as well as pressures in the pipes, stagnant areas, and slow sections of pipe, as well as leakage and backflow. These are only a few of the environmental uses for nanosensors. Air quality and water quality/quantity measurements are the two most prevalent environmental disturbance sensing applications.

## 3. System Design

The proposed system mainly focuses on the identification of skin disease using convolutional artificial intelligence algorithm. In the proposed system, the input skin image is given as digital format, and there are some unwanted things, and in order to move the unwanted things, we are using preprocessing technique. This technique is improving the quality of the image. The dataset is already given and also preprocessed. The MLP-BPNN algorithm checks the given skin image in the dataset, and at last, it will display the output as normal or abnormal skin [20] (Figure 1).

The article "An Enhancement on Convolutional Artificial Intelligent Based Diagnosis for Skin Disease Using Nanotechnology Sensors" was retracted in 2023. Reasons: signs of a paper mill; suspected computer-generated content; unreliable results or conclusions; concerns about the data.

In this system, the digital format image is given as input image should be given. The input image is given as digital format [7]. There are some noises in that image such as hair and bubbles. In order to remove the unwanted things, we are using image preprocessing technique. Preprocessing is used to remove unwanted things.

The study converts the raw text into vectors using the process of vectorization, and this uses a function called CountVectorizer that converts the text into word count matrix, where the matrix produced is of sparse type.

This technique also improves the accuracy of the image. The dataset is already collected, and the dataset is also preprocessed. Then, the algorithm used here is convolutional artificial intelligence algorithm. This algorithm checks the given input image with the data in the dataset, and when both the images were matched, it will display the type of the skin disease [21].

### 3.1. Multilayered Perceptrons

A neural organization is a blend of fake neurons. The neurons are commonly assembled into layers. In a completely associated feed-forward multilayer organization, each yield of a layer of neurons is taken care of as contribution to every neuron of the following layer. Consequently, a few layers measure the first information, while some cycle information got from different neurons. Every neuron has various loads [10] equivalent to the quantity of neurons in the past layer. A multilayer network commonly incorporates three sorts of layers: an info layer, at least one concealed layer, and a yield layer. The info layer typically simply passes information along without adjusting it. The majority of the calculation occurs in the concealed layers. The yield layer changes the shrouded layer initiations over to a yield, for example, an order. A multilayer feed-forward organization within any event one concealed layer can work as a general approximator, for example, it can be developed to process practically any capacity. In this postulation, we will generally talk about completely associated networks [22] and convolutional networks. Convolutional networks use boundary sharing and have restricted associations contrasted with completely associated networks.

### 3.2. Backpropagation

A neural organization is prepared by choosing the loads of all neurons so the organization figures out how to surmised target yields from known data sources. It is hard to address the neuron loads of a multilayer network systematically [23]. The back-spread calculation gives a basic and successful answer for addressing the loads iteratively. The traditional rendition utilizes angle plunge as enhancement technique. Slope plunge can be very tedious and is not ensured to locate the worldwide least of mistake, however with appropriate arrangement (referred to in AI as hyper-boundaries) functions admirably enough in 23 practices. In the main period of the calculation, an information vector is spread forward through the neural organization [24].

The article "An Enhancement on Convolutional Artificial Intelligent Based Diagnosis for Skin Disease Using Nanotechnology Sensors" was retracted in 2023. Reasons: signs of a paper mill; suspected computer-generated content; unreliable results or conclusions; concerns about the data.

A convolutional artificial intelligence (CAI) is a special neural network model that uses perceptron and estimation for the examination, that is, classification of data. MLP-BPNN enables proper processing of image, and it finds its application in the field of natural language processing and medical fields [24]. The MLP-BPNN operates with the principle of feed-forward network, and it reduces the number of edges without affecting the nature of information. The image consisting of high dimensionality is processed easily using MLP-BPNN that enables the classification of edges in any type of image [25].

Once the results are obtained from the algorithms, the feedback of the predicted results either correctly predicted or incorrectly predicted is sent to the classifier in the form of feedback.

## 4. Results and Discussion

The software output and interpretation of the type of skin disease according to that disease datasets are included for the outcome processing. Confirmation bias is the desire to select just the datasets that support or confirm something you already know, rather than facts that would reveal something that runs opposite to established views. The consequence is data that is polluted because it was selected in a biased manner or because information that does not confirm the predetermined notion is tossed out.

### 4.1. Input Parameters

The input parameters are discussed over the results chapter. The proposed system will give expected outcomes with the constrained input parameters. Tensorflow and Keras tools are used to reduce the execution time of algorithms (Figure 2) (Table 1)

### 4.2. Software Output

The output of this paper can be executed in a python terminal. Once the image name is given as an input, it will predict the disease type with the help of trained datasets and produce the result as below.

The above Figure 3 shows that the type of skin disease as an output. It will display a python list with some values in it. In this paper, we have four classifications of skin diseases such as melanoma (I), nevus (II), psoriasis (III), and seborrheic keratosis (IV). In the above figure, the python list displays a value 1.0 (accurate) in the first position, and it means that the input image is related to the first classification of skin disease (melanoma).

The article "An Enhancement on Convolutional Artificial Intelligent Based Diagnosis for Skin Disease Using Nanotechnology Sensors" was retracted in 2023. Reasons: signs of a paper mill; suspected computer-generated content; unreliable results or conclusions; concerns about the data.

As the above image (2.jpg) is given as an input (Figure 4), the output is as shown in Figure 5.

The above Figure 5 shows that the type of skin disease as an output. In this paper, we have four classifications of skin diseases such as melanoma (I), nevus (II), psoriasis (III), and seborrheic keratosis (IV).

In the above figure, the python list displays a value 1.0 (accurate) in the fourth position, and it means that the input image is related to the fourth classification of skin disease.

Table 2 shows the results of accuracy, where the MLP-BPNN classifier performs with a higher rate of classifying the skin cancer images than the other existing machine learning classifiers. The results of the simulation are high for all test images than for other methods.

Table 3 shows the results of sensitivity, where the MLP-BPNN classifier performs with a higher rate of classifying the skin cancer images than the other existing machine learning classifiers. The results of the simulation are high for all test images than for other methods.

Table 4 shows the results of specificity, where the MLP-BPNN classifier performs with a higher rate of classifying the skin cancer images than the other existing machine learning classifiers. The results of the simulation are high for all test images than for other methods.

Table 5 shows the results of the F-measure, where the MLP-BPNN classifier performs with a higher rate of classifying the skin cancer images than the other existing machine learning classifiers. The results of the simulation are high for all test images than for other methods.

## 5. Conclusion and Future Enhancement

In this paper, diagnosis of skin disease type with the help of the MLP-BPNN algorithm is included in the proposed solution. Large numbers of people in the world have skin disease due to people's unconsciousness and the risk factors of skin disease. The main contribution of the work involves the collection of images from nanosensors, which is the state-of-art in the proposed model. The sensing of the skin for its chemical, physical, and biological conditions has improved the detection ability for optimal classification. Most of the people lying below the poverty line fall under this category. Most of these people cannot reach a doctor and do most outdoor activities because of a lack of money. Most do not care about skin disease. Hence, the necessity of predicting skin disease plays a major role in the process of diagnosis. The proposed method can efficiently and successfully predict skin disease. A skin disease prediction system will be developed by the MLP-BPNN algorithm. The prediction system may be faster, less computationally expensive, time-efficient, and produce results that are more accurate. The proposed system will help doctors to efficiently predict skin diseases in the initial stages for better treatment. Skin disease diagnosis system identifies and recognizes symptoms and diagnoses melanoma in its early stages. The diagnosis method includes both image processing and artificial intelligence with an accuracy of 97.8%. MLP-BPNNs provide performance in a higher manner than the existing classifier. MLP-BPNN achieves higher accuracy in classifying the images of skin disease; however, there exist several rooms for improvement. It is concluded that the main objective of this paper is to predict the type of skin disease easily and also help the dermatologist to diagnose the skin diseases at an early stage to avoid the loss of lives of the people.

The article "An Enhancement on Convolutional Artificial Intelligent Based Diagnosis for Skin Disease Using Nanotechnology Sensors" was retracted in 2023. Reasons: signs of a paper mill; suspected computer-generated content; unreliable results or conclusions; concerns about the data.

## Figures and Tables

**Figure 1:** Proposed model.

**Figure 2:** Image (1.jpg).

**Figure 3:** Output for Image (1.jpg).

**Figure 4:** Image (2.jpg).

**Figure 5:** Output for image (2.jpg).

**Table 1:** Image Processing System to differentiate normal and abnormal images using CNN model.

Parameter	Value
Image name (jpg)	1.jpg

**Table 2:** Accuracy.

Images	NB	MLP	FFNN	BPNN	MLP-BPNN
100	0.954	0.947	0.972	0.97	0.978
200	0.921464	0.914614	0.939076	0.937119	0.944947
300	0.89237	0.885668	0.909603	0.907688	0.915348
400	0.868708	0.86215	0.885571	0.883697	0.891191
500	0.84547	0.839053	0.861969	0.860136	0.867469

**Table 3:** Sensitivity.

Images	NB	MLP	FFNN	BPNN	MLP-BPNN
100	0.921464	0.914614	0.939076	0.937119	0.944947
200	0.89237	0.885668	0.909603	0.907688	0.915348
300	0.868708	0.86215	0.885571	0.883697	0.891191
400	0.84547	0.839053	0.861969	0.860136	0.867469
500	0.829646	0.823367	0.84579	0.843996	0.851171

**Table 4:** Specificity.

Images	NB	MLP	FFNN	BPNN	MLP-BPNN
100	0.908744	0.868626	0.895045	0.921464	0.923421
200	0.879923	0.840669	0.86652	0.89237	0.894284
300	0.85653	0.818121	0.843414	0.868708	0.870582
400	0.833553	0.795971	0.820721	0.84547	0.847303
500	0.817986	0.781213	0.805429	0.829646	0.831439

**Table 5:** F-measure.

Images	NB	MLP	FFNN	BPNN	MLP-BPNN
100	0.914614	0.891131	0.916571	0.93027	0.934184
200	0.885668	0.86269	0.887583	0.900986	0.904816
300	0.86215	0.839667	0.864024	0.877139	0.880886
400	0.839053	0.817054	0.840887	0.853719	0.857386
500	0.823367	0.801842	0.825161	0.837718	0.841305

## Data Availability

The datasets used and/or analyzed during the current study are available from the corresponding author on reasonable request.
